RETRACTED

# FEZF1-AS1 is a key regulator of cell cycle, epithelial–mesenchymal transition and Wnt/β-catenin signaling in nasopharyngeal carcinoma cells

**DOI:** 10.1042/BSR20180906

**Published:** 2019-01-08

**Authors:** Yunzhou Cheng

**Affiliations:** Department of Pathology, People’s Hospital of Xintai City, Xintai City, Shandong Province 271200, China

**Keywords:** cell cycle, EMT, FEZF1-AS1, nasopharyngeal carcinoma, Wnt/β-catenin signaling

## Abstract

Background: Accumulating studies discloses that long non-coding RNAs (lncRNAs) serve important roles in human tumorigenesis, including nasopharyngeal carcinoma (NPC). The purpose of the present study was to determine the role of lncRNA FEZF1-AS1 in NPC.

Materials and methods: The expression levels of FEZF1-AS1 in NPC tissues and cell lines were detected by RT-qPCR analysis. MTT assay was performed to investigate the proliferation of NPC cells *in vitro*, whereas the migration and invasion of NPC cells were determined by wound healing assay and transwell assay. A nude mouse tumor model was established to study the role of FEZF1-AS1 in NPC tumorigenesis *in vivo*. The expression levels of proteins were detected by Western blot assay.

Results: The results showed that FEZF1-AS1 expression was increased in the NPC tissues and cell lines, and the higher expression of FEZF1-AS1 was closely associated with poor prognosis of NPC patients. We further observed that knockdown of FEZF1-AS1 inhibited the proliferation of NPC cells *in vitro* and suppressed NPC xenograft growth *in vivo* through inducing G2/M cell cycle arrest. The migratory and invasive abilities of NPC cells were also reduced upon FEZF1-AS1 knockdown. Moreover, we demonstrated that inhibition of FEZF1-AS1 remarkably suppressed epithelial–mesenchymal transition (EMT) and reduced β-catenin accumulation in nucleus in NPC cells.

Conclusions: Collectively, we showed that FEZF1-AS1 might be a key regulator of cell cycle, EMT and Wnt/β-catenin signaling in NPC cells, which may be helpful for understanding of pathogenesis of NPC.

## Introduction

Nasopharyngeal carcinoma (NPC) is a rare malignancy in most parts of the world but is common in China [1]. Annually, over 60,000 new cases of NPC were found in China [2]. Currently, the 5-year survival rate of NPC patients remains at 50–70% [3]. The development of NPC involves multiple genetic and epigenetic abnormalities [4]. Therefore, it is of critical importance to understand the molecular etiopathogenesis underlying NPC progression, which may help for the improvement of NPC diagnosis and treatment.

Long non-coding RNAs (lncRNAs) are a recently characterized class of non-protein coding RNA transcripts containing more than 200 nucleotides [5]. Emerging evidence showed that lncRNAs serve as tumor suppressors or oncogenes in cancer development [6]. For example, as a well-known member of lncRNAs, FEZ family zinc finger 1 antisense RNA 1 (FEZF1-AS1), mapped to 7q31.32 genomic region, is reported to be overexpressed in multiple human cancers, including colorectal carcinoma [7], osteosarcoma [8] and lung adenocarcinoma [9]. However, up to now, limited studies have determined the biological role of FEZF1-AS1 in NPC.

RETRACTED

In the present study, we examined the expression of FEZF1-AS1 in human NPC tissues and cell lines and explored its roles in regulating the malignant phenotypes of NPC cells.

## Materials and methods

### Patients and tissue samples

NPC tissues were collected from 71 patients with NPC who underwent surgery at People’s Hospital of Xintai City (Shandong, China). These patients did not receive any anticancer therapies before surgery. The demographic data and clinicopathological characteristics of these NPC patients were listed in Table 1. TNM staging was performed according to the 7th Edition of the AJCC/UICC Cancer Staging Manual. Normal nasopharyngeal epithelial tissues were collected from 10 healthy people. The tissue samples were snap-frozen in liquid nitrogen and stored at −80°C for further experiments. The Ethics Committee of People’s Hospital of Xintai City approved the present study procedure, and written informed consent was obtained from all participants.

**Table 1:** Correlation between FEZF1-AS1 expression and clinicopathological characteristics of NPC patients (*n*=71)

Characteristics	Total number (*n*=71)	FEZF1-AS1 expression		*P* value
		Low (*n*=39)	High (*n*=32)	
Age (years)				0.201
≤45	37	23	14	
>45	34	16	18	
Gender				0.637
Male	49	26	23	
Female	22	13	9	
EBV DNA copy				0.762
≤4000	28	16	12	
>4000	43	23	20	
TNM stage				0.060
I-II	27	11	16	
III-IV	44	28	16	
Distant metastasis				0.018
Yes	25	9	16	
No	46	30	16	

### Cell culture and transfection

A panel of NPC cell lines (6-10B, 5-8F, HNE1, CNE1 and CNE2) and the immortalized normal nasopharyngeal epithelial cell line (NP69) were cultured in Dulbecco’s Modified Eagle’s Medium (Thermo Fisher Scientific, Inc., Waltham, MA, U.S.A.) supplemented with 10% fetal bovine serum (FBS; Invitrogen, Carlsbad, CA, U.S.A.) and 1% penicillin/streptomycin in a humidified atmosphere containing 5% CO_2_.

The siRNA targeting FEZF1-AS1 (si-FEZF1-AS1) and negative control siRNA (si-NC) were constructed and synthesized by Ribobio (Guangzhou, China). Full-length sequences of FEZF1-AS1 were amplified by PCR and inserted into pcDNA3.1 vector (Realgene, Shanghai, China) to gain the FEZF1-AS1-overexpression plasmid. An empty vector served as a negative control. Transfection was achieved by using Lipofectamine 2000 (Invitrogen) according to a protocol provided by the manufacturer. After 48 h, transfection efficiency was detected by RT-qPCR analysis.

RETRACTED

### RNA extraction and RT-qPCR analysis

Total RNA was extracted from tissues and cells using TRIzol (Invitrogen). RNA was reversed into cDNA using the PrimeScript™ RT reagent kit (Takara, Dalian, China). qPCR analysis was then performed using SYBR® Premix Ex Taq™ II (TaKaRa) on an iCycler iQ™ Real-Time PCR Detection System (Bio-Rad Laboratories, Hercules, CA, U.S.A.). The data were calculated using 2^−ΔΔ*C*^_t_ method [10], and GAPDH was used as the endogenous control. The primers were designed as follows: FEZF1-AS1 forward, 5′-AGGGGATCGACGAGTTGAGA-3′ and reverse, 5′-TTGTCCCCGAGTCATTGGTG-3′; GAPDH, forward primer: 5′-CGACTTATACATGGCCTTA-3′ and reverse primer: 5′-TTCCGATCACTGTTGGAAT-3′. Each experiment was performed in triplicate.

### Western blot analysis

Total protein was extracted using radioimmunoprecipitation-assay buffer (Beyotime, Haimen, China). The nuclear and cytosolic fractions were prepared using the NE-PER Nuclear and Cytoplasmic Extraction Kit (Thermo Fisher Scientific). Equal amount of proteins (40 μg) was separated by sodium dodecyl sulfate-polyacrylamide gel electrophoresis and then electrophoretically transferred to polyvinylidene difluoride membranes (Millipore, Billerica, MA, U.S.A.). Next, the membranes were blocked with 5% skim milk and incubated with primary antibodies overnight at 4°C, followed by incubation with appropriated horseradish peroxidase-conjugated secondary antibodies. After washes, the bands were visualized with an enhanced chemiluminescence system (Pierce Biotechnology, Rockford, IL, U.S.A.), with GAPDH or Lamin B serving as a loading control. Each experiment was performed in triplicate.

### MTT assay

Cell proliferation was detected by 3-(4,5-dimethylthiazol-2-yl)-2,5-diphenyltetrazolium bromide (MTT) assay. In brief, after transfection, 2000 cells were seeded in a 96-well culture plate. At the indicated time points, 20 μl MTT (5 mg/ml; Sigma, St. Louis, MO, U.S.A.) was added to each well. After additional 4 h, 150 μl of DMSO was added into each well. Once the insoluble crystals were completely dissolved, the absorbance was detected at the wavelength of 570 nm using a spectrophotometric plate reader. Each experiment was performed in triplicate.

### Cell cycle analysis

Briefly, cells were washed with PBS three times and fixed with 80% ethanol. Then, cells were incubated with RNase A and stained with 20 μg/ml PI using the Cycle TEST PLUS DNA Reagent Kit (BD Biosciences, San Jose, CA, U.S.A.) at room temperature for 20 min. The percentages of cells in G0/G1, S and G2/M phase were analyzed by flow cytometry (BD Biosciences) and compared. Each experiment was performed in triplicate.

RETRACTED

### Wound healing assay

For wound healing assay, cells were seeded in six-well plates and subjected to serum starvation in serum-free medium for 24 h. Then, a sterilized 200 μl pipette tip was used to make an artificial wound in the confluent cell monolayer. Images were captured at 0, 24 and 48 h following the initial scratch. Each experiment was performed in triplicate.

### Transwell assay

In this assay, after transfection, 2 × 10^4^ cells suspended in 200 μl of serum-free medium were seeded into the upper chamber of each transwell (8 μm pore size, BD Biosciences), which was coated with or without Matrigel (BD Biosciences). About 600 μl medium containing 10% FBS was added to the lower chamber. After incubation for 24 h, the cells remaining on the upper membrane were removed using cotton swabs, and the cells on the lower membrane surface were fixed in methanol, stained with 1% Crystal Violet and counted under a light microscope with a magnification of ×200. Each experiment was performed in triplicate.

### Dual luciferase reporter assay

Cells were plated in 24-well plates and cotransfected with pcDNA3.1 vector, TOP Flash or FOP Flash reporter (Millipore, Temecula, CA, U.S.A.) and pRL-TK plasmids (Millipore) using Lipofectamine 2000. The luciferase signals were measured 48 h after transfection by using the Dual Luciferase Reporter Assay Kit (Promega). Each experiment was performed in triplicate.

### Animal studies

Ten BALB/c athymic nude mice (male 4–5 weeks old), obtained from Shanghai Laboratory Animals Center (Shanghai, China), were randomized to two groups (*n* = 5/group). A total volume of 200 μl of 1 × 10^6^ 5-8F cells stably transfected with sh-FEZF1-AS1 or sh-NC were inoculated subcutaneously into the left flanks of nude mice. The volumes of the tumors were measured every 3 days and calculated using the equation: volume = 0.5 × *W*^2^ × *L* (*W*, width; *L*, length). After 4 weeks, the mice were killed, and the tumors were removed for further analysis. All animal experiments were approved by the Ethics Committee of People’s Hospital of Xintai City.

### Statistical analysis

All statistical analyses were carried out using GraphPad Prism 6.0 software (GraphPad Software, San Diego, CA, U.S.A.) and SPSS 20.0 software (IBM, Chicago, IL, U.S.A.). Experimental results were expressed as mean ± standard deviation (SD) and analyzed by the Student’s *t*-test. The association between FEZF1-AS1 expression and clinicopathological features of NPC patients was evaluated using the chi-square test. Differences in the survival curve were evaluated using a log-rank test and drawn using Kaplan–Meier method. *P*-value <0.05 was considered statistically significant.

RETRACTED

## Results

### FEZF1-AS1 is up-regulated in NPC tissues and cell lines

First, as shown in Figure 1A, FEZF1-AS1 expression in NPC tissues was remarkably increased, compared with normal nasopharyngeal epithelial tissues. According to the average value of FEZF1-AS1 expression (2.58), the NPC patients were allocated into high FEZF1-AS1 expression group (>median; *n*=32) and low FEZF1-AS1 expression group (<median; *n*=39), and as summarized in Table 1, FEZF1-AS1 expression was closely correlated with distant metastasis (*P*=0.018) of NPC patients. In addition, high expression of FEZF1-AS1 was also significantly correlated with poor overall survival and disease-free survival of NPC patients (Figure 1B,C). To further confirm the up-regulation of FEZF1-AS1 in NPC, we measured its expression in a panel of NPC cell lines, and the results showed that five NPC cell lines expressed higher levels of FEZF1-AS1 than NP69 cells (Figure 1D). Among the five NPC cell lines, FEZF1-AS1 expressed highest in 5-8F cells and lowest in HNE1 cells, therefore these two cells were chosen for further study.

**Figure 1:** FEZF1-AS1 is up-regulated in NPC tissues and cell lines (**A**) RT-qPCR analysis of FEZF1-AS1 expression in the NPC tissues and normal nasopharyngeal epithelial tissues. (**B** and **C**) Kaplan–Meier analysis of overall survival and disease-free survival in 71 NPC patients according to FEZF1-AS1 expression. (**D**) RT-qPCR analysis of FEZF1-AS1 expression in a panel of NPC cell lines. Data are presented as the mean ± SD from three independent experiments *in vitro*. *P<0.05 versus NP69 cells.

### FEZF1-AS1 promotes NPC cell proliferation and cell cycle arrest

To determine the biological role of FEZF1-AS1 in NPC, FEZF1-AS1 was knocked down in 5-8F cells and overexpressed in HNE1 cells. After 48 h post-transfection, we confirmed that the transfection was successful (Figure 2A). The results of MTT assay indicated that the proliferation was suppressed remarkably in si-FEZF1-AS1-transfected 5-8F cells, whereas HNE1 cells with FEZF1-AS1 overexpression showed a significant promotion of proliferation (Figure 2B). Cell cycle arrest is a hallmark of restrained cell proliferation [11], therefore we subsequently checked whether the oncogenic role of FEZF1-AS1 is associated with induction of cell cycle arrest in NPC cells. As shown in Figure 2C, knockdown of FEZF1-AS1 significantly induced G0/G1 cell arrest in 5-8F cells, and the number of HNE1 cells in the S phase was increased following FEZF1-AS1 overexpression. Moreover, we observed that p21 expression was increased, whereas Cyclin D1 expression was decreased after FEZF1-AS1 knockdown in 5-8F cells, and FEZF1-AS1 overexpression had the opposite effects on the expression levels of these proteins in HNE1 cells (Figure 2D).

RETRACTED

**Figure 2:** FEZF1-AS1 promotes NPC cell proliferation and cell cycle arrest (**A**) The transfection efficacy was verified by RT-qPCR analysis. (**B**) The proliferation of 5-8F and HNE1 cells after transfection was detected by MTT assay. (**C**) The cell cycle distribution of 5-8F and HNE1 cells after transfection was detected by flow cytometric analysis. (**D**) The expression levels of p21 and Cyclin D1 in 5-8F and HNE1 cells after transfection were detected by Western blot analysis. Data are presented as the mean ± SD from three independent experiments *in vitro*. *P<0.05 versus si-NC-transfected 5-8F cells or empty vector-transfected HNE1 cells.

### Knockdown of FEZF1-AS1 suppresses NPC tumorigenesis *in vivo*

Next, we investigated the effects of FEZF1-AS1 on NPC tumorigenesis *in vivo*. We observed that the growth of tumors in the sh-FEZF1-AS1 group was significantly slower than that in the sh-NC group (Figure 3A), and after 4 weeks, the average weight of tumors in the sh-FEZF1-AS1 group was significantly lighter than that in the sh-NC group (Figure 3B). Furthermore, as shown in Figure 3C,D, p21 expression was increased, whereas the expression levels of FEZF1-AS1 and Cyclin D1 were reduced in the xenograft tissues derived from sh-FEZF1-AS1-transfected cells.

**Figure 3:** Knockdown of FEZF1-AS1 suppresses NPC tumorigenesis *in vivo* (**A**) Tumor volume growth curves were plotted. (**B**) The average tumor weight in each group was shown. (**C**) RT-qPCR analysis of FEZF1-AS1 expression in the xenograft tissues. (**D**) The expression levels of p21 and Cyclin D1 in the xenograft tissues were detected by Western blot analysis. Data are presented as the mean ± SD (*n* = 5/group). *P<0.05 versus sh-NC group.

### FEZF1-AS1 promotes NPC cell migration and invasion

In wound healing assay, we found that 5-8F cells transfected with si-FEZF1-AS1 migrated more slowly than those transfected with si-NC, and on the other hand, the migratory ability of HNE1 cells became much stronger upon FEZF1-AS1 overexpression (Figure 4A). Moreover, the results of transwell assay indicated that FEZF1-AS1 knockdown diminished the migratory and invasive abilities of 5-8F cells, whereas overexpressed FEZF1-AS1 significantly promoted the migration and invasion of HNE1 cells (Figure 4B).

**Figure 4:** FEZF1-AS1 promotes NPC cell migration and invasion (**A**) The migratory abilities of 5-8F and HNE1 cells after transfection were detected by wound healing assay. (**B**) The migration and invasion of 5-8F and HNE1 cells after transfection were detected by transwell assay. Data are presented as the mean ± SD from three independent experiments *in vitro*. *P<0.05 versus si-NC-transfected 5-8F cells or empty vector-transfected HNE1 cells.

RETRACTED

### FEZF1-AS1 induces EMT in NPC cells

EMT is critical for migration and invasion of cancer cells, and thus we explored whether FEZF1-AS1 exerts effects on EMT of NPC cells. As shown in Figure 5, E-cadherin expression was significantly increased while the expression levels of N-cadherin and Vimentin were obviously decreased in 5-8F cells following FEZF1-AS1 knockdown. Besides, FEZF1-AS1 overexpression significantly reduced the expression of E-cadherin and elevated the expression of N-cadherin and Vimentin in HNE1 cells.

**Figure 5:** FEZF1-AS1 induces EMT in NPC cells The expression levels of E-cadherin, N-cadherin and Vimentin in 5-8F and HNE1 cells after transfection were detected by Western blot analysis. Data are presented as the mean ± SD from three independent experiments *in vitro*. *P<0.05 versus si-NC-transfected 5-8F cells or empty vector-transfected HNE1 cells.

### FEZF1-AS1 activates Wnt/β-catenin signaling in NPC cells

Wnt/β-catenin signaling also serves a crucial role in NPC. As expected, we observed that FEZF1-AS1 knockdown decreased, whereas FEZF1-AS1 overexpression increased the luciferase activity of TOP/FOP report in NPC cells (Figure 6A). In addition, Western blot analysis showed that FEZF1-AS1 knockdown decreased, whereas FEZF1-AS1 overexpression increased the nuclear β-catenin accumulation in NPC cells (Figure 6B).

**Figure 6:** FEZF1-AS1 activates Wnt/β-catenin signaling in NPC cells (**A**) Dual luciferase reporter assay using TOP/FOP flash vectors was performed to determine the activity of Wnt/β-catenin signaling in 5-8F and HNE1 cells after transfection. (**B**) The expression levels of β-catenin in the nuclear and cytosolic fractions of 5-8F and HNE1 cells after transfection were detected by Western blot analysis. Data are presented as the mean ± SD from three independent experiments *in vitro*. *P<0.05 versus si-NC-transfected 5-8F cells or empty vector-transfected HNE1 cells.

## Discussion

The molecular mechanisms underlying NPC are very complicated and still poorly understood. Recent studies indicated that dysregulation of lncRNA expression is implicated in the development of NPC by functioning as tumor suppressors or oncogenes [12]. For example, lncRNA LINC0086 serves as a tumor suppressor in NPC [13], and lncRNA-n326322 promotes the proliferation and invasion of NPC cells [14]. The present study examined the biological role of lncRNA FEZF1-AS1 in human NPC.

RETRACTED

Our results indicated that FEZF1-AS1 was up-regulated in both NPC cell lines and clinical tissue samples. High FEZF1-AS1 expression is also closely correlated with aggressive tumor progression and unfavorable prognosis of NPC patients. Cancer cells express many malignant phenotypes. Further functional assays demonstrated that knockdown of FEZF1-AS1 significantly suppressed cell proliferation, migration and invasion *in vitro*, and inhibited NPC xenograft growth in rodent models. These findings suggested that FEZF1-AS1 functions as an oncogene in the tumorigenesis and progression of NPC.

NPC shows highly invasive and metastatic features [15]. Epithelial–mesenchymal transition (EMT) is critical for cancer cells to acquire metastatic ability. EMT is featured by a loss of epithelial markers, including E-cadherin, and the acquisition of mesenchymal proteins, including N-cadherin and Vimentin [16]. In non-small cell lung cancer and hepatocellular carcinoma, down-regulation of FEZF1-AS1 suppressed EMT process [17,18]. EMT is also closely related to the invasion and metastasis of NPC. Herein we found that FEZF1-AS1 up-regulated N-cadherin, Vimentin and down-regulated E-cadherin in NPC cells, indicating that FEZF1-AS1 might be a driver for EMT in NPC.

Abnormal activation of Wnt/β-catenin signaling is implicated in many types of cancers, including NPC [19]. As a central mediator of Wnt/β-catenin signaling, β-catenin also serves as a component of the cadherin complex, which controls cell–cell adhesion [20]. Several studies showed that Wnt/β-catenin signaling is a critical pathway to activate EMT [21]. Herein we believed that FEZF1-AS1 enhanced β-catenin entry of nucleus, which might be an important step in the induction of EMT in NPC. The molecular mechanisms by which FEZF1-AS1 exerts its oncogenic properties in NPC merit further investigation.

Taken together, our findings showed that lncRNA FEZF1-AS1 enhanced cell proliferation, migration and invasion capacities in NPC cells through inducing EMT and activating Wnt/β-catenin signaling. We suggested that FEZF1-AS1 serves as an oncogene in NPC, and we believed our findings might inject some new vitalities into the identification of therapeutic targets for NPC.

## Abbreviations

EMT: epithelial–mesenchymal transition
lncRNA: long non-coding RNA
NPC: nasopharyngeal carcinoma
